# Adhesive Bond Integrity of Experimental Zinc Oxide Nanoparticles Incorporated Dentin Adhesive: An SEM, EDX, *μ*TBS, and Rheometric Analysis

**DOI:** 10.1155/2022/3477886

**Published:** 2022-08-10

**Authors:** Yasser F. Alfaawaz, Renad Alamri, Fatimah Almohsen, Sana Shabab, Mai M. Alhamdan, Khold Al Ahdal, Imran Farooq, Fahim Vohra, Tariq Abduljabbar

**Affiliations:** ^1^Department of Restorative Dental Sciences College of Dentistry, King Saud University, Riyadh, Saudi Arabia; ^2^Dental Intern, College of Dentistry, King Saud University, Riyadh, Saudi Arabia; ^3^Department of Prosthetic dental sciences, College of Dentistry, King Saud University, Riyadh, Saudi Arabia; ^4^Faculty of Dentistry, University of Toronto, Toronto, ON, Canada M5G 1G6; ^5^Department of Prosthetic Dental Science, College of Dentistry, King Saud University 11545, Saudi Arabia

## Abstract

**Objective:**

Our study is aimed at preparing an experimental adhesive (EA) and assessing the influence of adding 5-10 wt.% concentrations of zinc oxide (ZnO) nanoparticles on the adhesive's mechanical properties.

**Methods:**

Field emission scanning electron microscopy (FESEM) and energy dispersive X-ray (EDX) spectroscopy were employed to investigate the morphology and elemental distribution of the filler nanoparticles. To examine the adhesive properties, microtensile bond strength (*μ*TBS) testing, an investigation of the rheological properties, degree of conversion (DC), and analysis of the interface between the adhesive and dentin were carried out.

**Results:**

The SEM micrographs of ZnO nanoparticles demonstrated spherical agglomerates. The EDX plotting confirmed the incidence of Zn and oxygen (O) in the ZnO nanoparticles. The highest *μ*TBS was observed for nonthermocycled (NTC) 5 wt.% ZnO group (32.11 ± 3.60 MPa), followed by the NTC-10 wt.% ZnO group (30.04 ± 3.24 MPa). Most of the failures observed were adhesive in nature. A gradual reduction in the viscosity was observed at higher angular frequencies, and the addition of 5 and 10 wt.% ZnO to the composition of the EA lowered its viscosity. The 5 wt.% ZnO group demonstrated suitable dentin interaction by showing the formation of resin tags, while for the 10 wt.% ZnO group, compromised resin tag formation was detected. DC was significantly higher in the 0% ZnO (EA) group.

**Conclusion:**

The reinforcement of the EA with 5 and 10 wt.% concentrations of ZnO nanoparticles produced an improvement in the adhesive's *μ*TBS. However, a reduced viscosity was observed for both nanoparticle-reinforced adhesives, and a negotiated dentin interaction was seen for 10 wt.% ZnO adhesive group. Further research exploring the influence of more filler concentrations on diverse adhesive properties is recommended.

## 1. Introduction

Adhesives in dentistry are bonded to either enamel or dentin, enamel being apt for adhesive bonding as it is predominantly inorganic [1]. Dentin is a collagenous tissue that helps anchor resin-based dental materials with the tooth structure; however, the gradual degradation of the resin-dentin bond remains a fundamental concern in adhesive dentistry [2]. This biodegradation causes microleakage, which assists secondary caries development, leading to restoration failure [3]. Dentin adhesives can play a part in preventing the degradation of the resin-dentin interface by providing adequate sealing [4]. A durable adhesive-dentin bond augments the longevity of the restoration, but the quality of this bond is extremely reliant on the composition of the adhesives [5]. The composition of dentin adhesives has been improved in the last few decades to improve their bonding capabilities [6]. This compositional change has improved the quality of the chemical bonds formed between adhesive and hydroxyapatite (HA) minerals of enamel or dentin [7]. However, despite the augmentations in the adhesive's composition, an adhesive that provides an ideal seal and optimum properties is still being pursued [8].

Nanotechnology is an emerging field, and it can be applied to dentistry to improve the diagnosis, treatment, and properties of various materials [9]. Nanofiller addition in the adhesive composition is an exciting prospect as it can enhance its bond strength and resin tag forming capability and reduces polymerization shrinkage [5]. The nanosize of these filler particles potentially helps them to enjoy superior chemical reactivity (due to a large surface area to mass ratio) and thus possibly entail strong mechanical and antibacterial properties [10, 11]. However, these improvements in mechanical and antibacterial properties are also dependent on the type of nanofiller being used in the adhesive. Previously, researchers have incorporated nanofillers in the adhesive based on bioactive glasses, HA, amorphous calcium phosphate (ACP), graphene oxide (GO), and zinc chloride (ZnCl_2_) [12]. Although nanofiller groups have revealed promising results, the quest to find a nanofiller group that can optimally improve various adhesive properties still endures.

Zn is a natural microelement in the body that is considered to be important as it contributes to various life activities by being part of different macromolecules and enzymes [13]. Zn has enticed particular attraction in dentistry owing to its known antibacterial properties [14]. Also, during the carious process, endogenous matrix metalloproteinases (MMPs) can cause degradation of dentin collagen and collapse of the adhesive interface during restoration [15]. Zn is known to be a MMP inhibitor, and it performs this function by binding to the collagen-sensitive cleavage sites of MMPs [16]. This certifies that for clinical dental applications, nanoparticles based on Zn could be useful in preventing collagen degradation in dentin. In addition, oxides of Zn (ZnO) have also been produced and are shown to be biocompatible, stable, low in toxicity, and cost-effective [17]. These beneficial characteristics make ZnO nanoparticles an ideal candidate to be integrated as a filler in dentin adhesives. Previously, ZnO quantum dots were added as fillers in the experimental adhesive (EA), and it was reported that ZnO-containing adhesive demonstrated a stable dentin-adhesive interface (even after 6-month post-treatment) when compared with the control adhesive [18]. In another study, the inclusion of ZnO in the adhesive enhanced its antimicrobial properties without affecting its physical and chemical functionality [19]. Similar results were reported by Saffarpour et al., and it was demonstrated that the addition of ZnO nanoparticles improves antimicrobial properties of the adhesives without impacting their bond strength [20]. Considering the beneficial properties of ZnO nanoparticles, the decision to incorporate them in the polymer-based adhesive in the current study was taken.

Therefore, the current study is aimed at including ZnO nanoparticles in the EA and exploring the impact of incorporation on its rheological properties, microtensile bond strength (*μ*TBS), and dentine interface. This study's null hypothesis (H_o_) was that ZnO-containing adhesive would behave similar to the EA (without nanofillers) in terms of the improvement of the above-mentioned properties.

## 2. Materials and Methods

The current study was approved by the institute's ethics committee, and all the protocols were strictly followed. We obtained teeth for the bonding experiments from the dental department, and caries and restoration free teeth were utilized.

### 2.1. Acquisition of ZnO Nanoparticles, Preparation of the EA, and Their Amalgamation

ZnO nanoparticles used in this study were sourced commercially (Merck, Darmstadt, Germany). Preparation of the EA was accomplished, as described previously [21]. Briefly, we incorporated monomers, encompassing BisGMA, TEGDMA, HEMA, and ethyl dimethyl-amino benzoate and camphor-quinone (Esstech Inc., Essington, PA, USA). The details can be obtained from a previous study [21]. The mixture was formulated using a flask, magnetic stirrer, and condenser (Bruker, Tokyo, Japan). The adhesive was kept in a dark sealed container. This adhesive was regarded as EA. Two concentrations of ZnO nanoparticles (5 and 10 wt.%) were then added to the EA separately to produce three adhesives: EA (control-0% ZnO), 5 wt.% ZnO, and 10 wt.% ZnO adhesive. These three adhesives were sonicated in a centrifuge and stored at 4°C.

### 2.2. Filler Nanoparticle Characterization

To characterize the filler nanoparticles, we employed field emission scanning electron microscopy (FESEM). ZnO nanoparticles were placed on aluminum stubs, sputter-coated with gold, and viewed in an SEM (FEI Quanta 250, Scanning Electron Microscope, OR, USA), as suggested in previous study [21]. The SEM was operated to observe morphological characteristics of ZnO nanoparticles. Energy dispersive X-ray (EDX) spectroscopy was employed for elemental distribution analysis of the ZnO nanoparticles.

### 2.3. Characterization of the Adhesives

The characterization of the adhesives in our study was carried out via multiple techniques. First, adhesives were assessed for rheology with a rheometer (Anton Paar, Graz, Austria). The rheology of these adhesives was appraised utilizing similar protocol (rotation mode) as used by Al-Saleh et al. [22]. The adhesive specimens were evaluated using angular frequencies ranging between 0.1 and 100 rad/s at 25°C, as formerly suggested by Al-Saleh et al. [22]. Further characterization of the adhesives was carried out by assessing their microtensile bond strength (*μ*TBS) and evaluating the integrity of the resin-dentin interface, in line with previous studies [21, 22] as explained below.

### 2.4. Specimen Preparation for Bonding, Analysis of *μ*TBS, and Failure Modes

Seventy-five teeth were mounted in ortho resin (Opti-Cryl, South Carolina, Columbia) with a 15 mm (height) segment of polyvinyl. Their dentin was exposed using a handpiece (Dental Corp., Biberach, Germany) with a diamond disc. The three study groups, 0% ZnO, 5 wt.% ZnO, and 10 wt.% ZnO, received 25 teeth each. The dentin of these teeth was washed with distilled water, followed by their air drying and etching with 36% phosphoric acid (DeTrey conditioner, Dentsply, PA, USA). Samples were etched for 15 seconds. A microbrush was employed to apply adhesives onto the dentin of these teeth for 5 s. The first smearing of the adhesives onto the dentinal surface was trailed by air thinning for 3 s, followed by another application of the adhesive layer (5 s). The curing of the adhesives was performed for 20 seconds with a curing light (Bluephase, Ivoclar, Vivadent, Amherst, New York, USA), and the distance between the light and the adhesive was maintained at 10 mm. After curing, a polymer composite layer (Multicore Flow; Ivoclar, Vivadent, Amherst, New York, USA) of 2 mm was placed over each tooth and then polymerized using the same parameters as mentioned for the adhesive curing. Twenty samples in each group were designated for the *μ*TBS test, and five were used for resin-dentin interface analysis. Among the *μ*TBS samples, half of the bonded samples were thermocycled (TC) before the test inside a thermocycler (THE-1100, SD Mechatronik GmbH, Germany). In this study, 10,000 cycles in water baths were used for the aging of the samples with 5-55°C temperature. The time for which each sample was exposed to water for aging was 30 s, and a dwell time of 5 s. The remaining ten samples remained nonthermocycled (NTC) and were stored in deionized water. The TC samples were also shifted to deionized water after the aging experiments were completed.

The bond failure types were assessed with a digital microscope (Hirox KH 7700, Tokyo, Japan). The category of failure types was adhesive, cohesive, and/or mixed, and it was dependent on the site where the fracture was observed.

### 2.5. Assessment of the Resin-Dentin Interface

The bonded tooth samples for the assessment of resin-dentin interface were sectioned with a slow-speed isomet saw (Isomet 2000 Precision saw, Lake Bluff, IL, USA). The sectioning assisted in the formation of 1 × 1 mm beams. A maximum of six bonded beams were produced and tested for each tooth, resulting in a total of sixty beams in each group. The microtensile bond strength test was performed at constant load of 100 N (load cell) and a crosshead speed of 0.5 mm/min using a universal testing machine (Instron, 5969, Testing machine, Norwood, MA, USA). The FESEM was utilized to appraise the resin-dentin interface's integrity, and it was judged by resin tag formation. The methodology was adapted from previous studies [21, 22].

## 3. Degree of Conversion

The extent of double bond conversion was assessed using FTIR, and a standard protocol was utilized to assess the degree of conversion (DC) [23]. The 0% ZnO, 5 wt.% ZnO, and 10 wt.% ZnO adhesives were applied on the spectroscope (Thermo Scientific Nicolet iS20 FTIR spectrometer, MA USA). Eight readings with each adhesive were performed, and a mean and standard deviation was calculated. The area under peaks of the aliphatic (at 1638 cm^−1^) and aromatic (1608 cm^−1^) C=C were calculated before and after polymerization (60 s). For observing the DC, assessment formula and evaluations were adopted from previous study [23].

### 3.1. Statistical Analysis

The *μ*TBS results were gathered, computed on an excel sheet, and then evaluated using Statistical Package for the Social Sciences (SPSS-20.0, IBM, Chicago, IL, USA). The Kolmogorov–Smirnov test was applied to check the normality of the data. Upon observing nonparametric distribution, the ANOVA and post hoc multiple comparison tests were used to equate the means and SD of different adhesive groups. The level of significance was set at 1%.

## 4. Results

### 4.1. Outcomes of the Characterization of Filler Nanoparticles

Morphologically, the ZnO nanoparticles demonstrated spherical to irregularly shaped polygonal crystals on the SEM micrograph (Figure 1). These nanoparticles were seen without any sharp angles or edges and agglomerating with each other. The particle size of our filler when observed under an SEM ranged between 500 and 1000 nm. On EDX analysis, these filler nanoparticles confirmed the presence of Zn (Figure 1).

### 4.2. Outcomes of Rheological Assessment

The rheological evaluation of our three adhesives demonstrated that at higher angular frequencies, a gradual decrease in the viscosity was observed (Figure 2). Considering these results, it can be confirmed that our adhesives have shown non-Newtonian behavior (shear-thinning or pseudoplasticity). In the present study, the addition of 5 and 10 wt.% ZnO to the composition of the EA lowered its viscosity; however, this finding was not consistent, and the viscosities of all the adhesive groups intersected at higher frequencies (Figure 2).

### 4.3. Outcomes of the *μ*TBS and Failure Mode Investigation

The *μ*TBS results for the three adhesive groups (EA, 5 wt.% ZnO, and 10 wt.% ZnO) are shown in Table 1. For both NTC and TC, the highest *μ*TBS was obtained for 5 wt.% ZnO adhesive. In case of 5 wt.% ZnO, the *μ*TBS significantly dropped after TC (Table 1). The highest *μ*TBS (32.11 ± 3.60 MPa) was observed for NTC-5 wt.% ZnO followed by NTC-10 wt.% ZnO group (30.04 ± 3.24 MPa). The next highest *μ*TBS (29.63 ± 3.10 MPa) was perceived for TC-5 wt.% ZnO followed by TC-10 wt.% ZnO group (27.25 ± 3.71 MPa), while the EA presented the lowest *μ*TBS values for both NTC and TC samples (25.33 ± 3.40 and 24.70 ± 3.55 MPa, respectively (Table 1). The intergroup comparisons were significant (*p* < 0.01) when the *μ*TBS values of EA were matched with the other groups for both TC and NTC samples. The intragroup comparisons were only significant (*p* < 0.01) for 5 wt.% ZnO group when the NTC and TC samples were compared (Table 1).

The failure modes witnessed in our study are also presented in Table 1. The adhesive type interfacial failures were found to be most common in our study (ranging between 70 and 100%). The mixed type failures were found to be the next most common type of failures (ranging between 20 and 30%). None of the failures observed were of the cohesive type.

### 4.4. Outcomes of the Resin-Dentin Interface Assessment

The illustrative SEM micrographs displaying the interface between EA, 5 wt.% ZnO, and 10 wt.% ZnO adhesive groups and dentin are presented in Figures 3(a)–3(c). The EA (control) demonstrated appropriate resin tag formation and hybrid layer (Figure 3(a)). For the 5 wt.% ZnO adhesive group, comparable resin tag and hybrid layer formation were seen (Figure 3(b)). For the 10 wt.% ZnO group, that fewer resin tags were formed (as compared to the EA and 5 wt.% ZnO groups) (Figure 3(c)).

## 5. Degree of Conversion

The FTIR spectra of 0% ZnO, 2.5% ZnO, and 5% ZnO groups (cured and uncured) were recorded.  Figure 4 presents double bond conversion FTIR peaks for 5% ZnO adhesives. The DC was evaluated by estimating the differences in peak height ratio among absorbance strengths of aliphatic C═C peak (1638 cm^−1^) and standard inner peak of aromatic C═C (1608 cm^−1^) while polymerization. For DC analysis, the maximum DC was observed with 0% ZnO adhesive (68.24 ± 7.3) followed by 5% ZnO adhesive (42.91 ± 6.7) (Table 2). The least DC was shown in 10% ZnO adhesive (38.32 ± 6.3). DC was significantly higher in 0% ZnO adhesive compared to 5% and 10% ZnO specimens (*p* < 0.01). No statistically significant results (*p* > 0.01) were witnessed between DC values of 5% and 10% ZnO.

## 6. Discussion

Based on this study's findings, we partly reject the H_o_ as the two nanofiller-reinforced adhesives demonstrated higher bond strength compared to the EA. We also partially accept the H_o_ as the 5 wt.% ZnO and 10 wt.% ZnO adhesives revealed lower viscosity when matched with the EA. Several earlier studies have verified that the reinforcement of adhesives by the addition of bioactive inorganic filler nanoparticles can improve its mechanical properties [21, 24]. Related to medical and dental applications, ZnO nanoparticles have been largely investigated in the past for their antimicrobial potential [19, 25, 26]. There is a scarcity of studies in the literature, which have used ZnO nanoparticles to reinforce dentin adhesive's mechanical properties. Therefore, it was decided in this study to incorporate ZnO nanoparticles as filler in the composition of our EA and then assess the effect of their insertion on various properties of the EA.

The filler nanoparticles in this study revealed spherical to irregularly shaped agglomerated nanoparticles on the SEM micrograph (Figure 1). This finding is consistent with several previous studies that also demonstrated agglomeration of spherical-shaped ZnO nanoparticles on SEM micrographs [27, 28]. The morphology of ZnO nanoparticles could be altered with numerous factors, including temperature change [29] and stirring time during synthesis [30]. In the present study, ZnO was commercially acquired; hence, the reason for observing spherical-shaped agglomerated nanoparticles cannot be understood. The EDX mapping in this study verified the presence of only Zn and O inside the ZnO nanoparticles (Figure 2). This conforms to a previously published study, which demonstrated that EDX mapping of ZnO nanoparticles shows that the product is 100% composed of only Zn and O atoms [31].

Regarding rheological properties, it was noticed that all adhesives in our study demonstrated a reduced viscosity at higher angular frequencies (Figure 3). A previous study showed similar findings and reported that ZnO nanoparticles containing composites also displayed shear-thinning behavior [32]. Another similar study echoed our findings and reported that the adhesives containing nanoparticles show reduced viscosity at higher angular frequencies [33]. It should be taken into account that the rheological properties are unpredictable and they can be altered by several factors (including material's handling during preparation and experiments) [34].

Our results demonstrated that NTC-5 wt.% ZnO showed the highest bond strength followed by NTC-10 wt.% ZnO group. These findings are in line with a former study that has shown that the addition of nanoparticles based on the oxides of quasimetals in the adhesive improves their bond strength [35]. It is a known fact that MMPs in the dentin are exposed due to etching, and they degrade type 1 collagen fibers [36], which can directly impact the bond strength of the adhesive. Osorio et al. previously reported that Zn-based nanoparticles have an inhibitory effect on MMP activity [37]. Also, similar findings were reported by Gutiérrez et al. and demonstrated an anti-MMP activity associated with ZnO nanoparticles containing adhesive [38]. The release of ZnO nanoparticles from resin polymer matrix in its surrounding environment is considered as inevitable and obvious [39]. In addition, the ZnO nanoparticle release may amplify with increase in concentration of incorporated ZnO nanoparticles [39]. Therefore, it is possible that ZnO nanoparticles in our study prevented the denaturation of collagen fibers by reducing MMP activity, leading to the establishment of a stronger bond between the adhesive and dentin which was verified by increased *μ*TBS values for ZnO-reinforced adhesives. We also noticed that the bond strength values decreased when the filler concentration increased from 5 to 10 wt.%. ZnO is an opaque material that can obscure the pathway of curing light [40]. It was observed in the present study that an increase in the ZnO concentration may have blocked adequate conversion of monomers into polymers, hence causing 10 wt.% ZnO group to display reduced *μ*TBS values (although they were still higher than the EA). Another credible reason explaining this finding could be the agglomeration phenomenon [41], and it can escalate with an increasing filler concentration causing reduced bond strength, as observed for our 10 wt.% ZnO group. ZnO particles are known to react with the carbonyl, aromatic, amide N-H, and acidic groups in the adhesive and form zinc methacrylate and dimethacrylate [42]. In addition, the Zn nanoparticles may interact with urethane groups via surface hydroxyl group, hence making a strong bond [43]. Another trend observed for *μ*TBS results was that TC samples presented lower bond strength values compared to their NTC counterparts. Thermocycling is a suitable method to replicate *in vivo* aging in an *in vitro* environment [44]. Several previous studies have demonstrated that the aging of adhesive bonded tooth samples via thermocycling can cause a reduction in the bond strength [45], and our results agree with these studies. The majority of the failures in this study were found to be adhesive in nature. It is common to find these types of failures in adhesives when inorganic filler nanoparticles are integrated into their composition [36]. It should be kept in mind that dentin's wettability offers significant challenges in adhesive bonding [46] and can lead to these failures.

Adhesive penetration inside the dentinal tubules is desirable as it could form stronger adhesive-dentin bonds [1]. The SEM micrographs to evaluate adhesive-dentin interface analysis exhibited the presence of standard resin tags and dentin penetration for 5 wt.% ZnO group when compared with the EA. Previously, Gutiérrez et al. demonstrated that the inclusion of ZnO nanoparticles can improve dentin interaction of the adhesive (by improving the integrity of the hybrid layer) [47]. Our study findings are in agreement with their study as we also observed the presence of appropriate resin tags and hybrid layer formation. However, for 10 wt.% ZnO group, a compromised resin tag formation was observed. It is possible that in the present study, an increased filler concentration impacted adequate penetration of dentinal tubules to form resin tags.

Concerning the limitations of the present study, one major limitation was its *in vitro* nature. It should be kept in mind that the *in vivo* environment is vibrant and can offer numerous unanticipated challenges to the foreign material. Also, we observed a compromised resin tag formation when the filler content was increased. It is pertinent to mention that the Zn particles were not silanized in the present study; however, silanization is known to enhance the resin adhesion to inorganic fillers [48]. In addition, zinc is associated with matrix metalloproteinases- (MMP-) related collagen protection in the hybrid layer [47]; however, its (Zn) percentage correlation to MMP levels is not investigated in the present experiments. Therefore, further studies evaluating the influence of silanized Zn particles in dentin adhesive and its association with biological mediators in protecting dentin are recommended. Also, *in vivo* performance of these nanoparticle-reinforced adhesives should be evaluated. In the present study, the 0% ZnO adhesive showed higher DC as compared with 5% and 10% ZnO incorporated adhesives. Incorporation of nanoparticle fillers in polymeric adhesives has shown increase of the adhesive's bond strength and a decline in DC in previous studies [24, 49]. A possible explanation for decrease in DC on incorporation of ZnO particles is a reduction in curing light penetration through the adhesive medium for monomer to polymer conversion, thereby resulting in a loss of DC [50].

Our study's findings show potential for ZnO-reinforced adhesives for further assessments, as they performed superiorly to the controls by demonstrating higher *μ*TBS. A higher bond strength could improve longevity of the resin restoration which could not only be cost-effective for the patients but could also reduce potential damage to their teeth that could ensue during replacement of a failed resin restoration.

## 7. Conclusions

The addition of 5 wt.% ZnO nanoparticles improved the adhesive's mechanical properties (bond strength and dentin interaction). The 5 wt.% ZnO nanoparticles containing adhesives demonstrated the highest bond strength. In the 10 wt.% ZnO nanoparticles containing adhesive, although displayed a higher bond strength when compared with the EA, a compromised resin tag formation was observed for this adhesive group. The current findings could have implications for clinical dentistry as these ZnO-reinforced adhesives could potentially improve the longevity of the resin restorations. Further studies exploring the influence of more filler concentrations on other adhesive properties are recommended. Also, *in vivo* performance of these nanoparticle-reinforced adhesives should be evaluated.

## Figures and Tables

**Figure 1:** (a) High-magnification FESEM image of Zn oxide (ZnO) agglomerated particles of irregularly sized crystals, ranging from 500 nm to 1000 nm. (b) Representative EDX graph showing presence of Zn.

**Figure 2:** Rheological properties of the 0% ZnO (control), 5% ZnO, and 10% ZnO adhesives. Complex viscosity is presented for angular frequencies of 0.001 to 1000 rads/s.

**Figure 3:** FESEM images of resin-dentin interface showing (a) adhesive resin (AD), hybrid layer (HL), and normal resin tag (RT) formation in control samples (0% ZnO). (b) Normal resin tag formation and dentin penetration with 5% ZnO particle incorporated dentin adhesive. (c) RT formation and dentin penetration were compromised in 10% ZnO particle (few resin tags).

**Figure 4:** Typical double-bond conversion FTIR peaks before and after curing for 5% ZnO adhesives.

**Table 1:** Means and standard deviations for bond strength and failure modes among the study groups.

	*μ*TBS (MPa) (mean ± SD)			Failure mode analysis (%)		
Group (*n* = 10)	NTC	TC	*p* value^∗^	Adhesive	Cohesive	Mixed
0% ZnO	25.33 ± 3.40^aA^	—	<0.01	100	0	0
	—	24.70 ± 3.55^aA^		100	0	0
5.0 wt.% ZnO	32.11 ± 3.60^bA^	—		70	0	30
	—	29.63 ± 3.10^bB^		80	0	20
10.0 wt.% ZnO	30.04 ± 3.24^bB^	—		80	0	20
	—	27.25 ± 3.71^bB^		100	0	0

TC: thermocycling; NTC: no thermocycling; ZnO: zinc oxide. ^∗^ANOVA. Dissimilar lower case letters in the same column indicate statistical significance. Dissimilar capital letters in a row (same group) indicate statistical significance.

**Table 2:** Degree of conversion among the different study adhesives.

No.	Group name	DC (%)^∗^
1	0% ZnO	68.24 ± 7.3^A^
2	5% ZnO	42.91 ± 6.7^B^
3	10% ZnO	38.32 ± 6.3^B^

^∗^ANOVA. Dissimilar superscript capital alphabets denote significant difference among groups.

## Data Availability

Data is accessible from the corresponding author on request.
